# The Clinical Observation on PONV with the Intervention of Thumbtack Needles Combined with Chinese Medicine Ironing Therapy

This article has been retracted.

**DOI:** 10.1155/2022/2498995

**Published:** 2022-07-30

**Authors:** Bao-Lian Guo, Fang-Ping Lou

**Affiliations:** ^1^Department of Urology, Zhuji People's Hospital, Shaoxing, Zhejiang Province, China; ^2^Department of Orthopedics, Zhuji Hospital of Traditional Chinese Medicine, Shaoxing, Zhejiang Province, China

## Abstract

**Objective:**

This study aimed to analyze the clinical efficacy of the intervention of thumbtack needles (applicable to subcutaneous embedding) combined with Chinese medicine ironing therapy on postoperation nausea and vomiting (PONV).

**Methods:**

106 patients who scheduled elective surgery were enrolled and randomized into control group and experimental group, with 53 cases in each group. The control group received modern medication, while the experimental group was given thumbtack needles combined with Chinese medicine ironing therapy based on the control group. The PONV score, incidence rate, gastrointestinal hormone level, Functional Living Index-Emesis (FLIE), and General Comfort Questionnaire (GCQ) of the two groups were compared.

**Results:**

After treatment, the incidence of PONV and GCQ in the experimental group was observed to be remarkably lower than that in the control group (*P* < 0.05), while the levels of gastrointestinal hormones and the level in the FLIE of the experimental group were comparatively higher than those in the control group (*P* < 0.05).

**Conclusion:**

Thumbtack needles combined with Chinese medicine ironing therapy can be utilized to reduce the incidence of PONV, to improve the level of gastrointestinal hormones, and to improve the comfort and quality of patients' lives.

## 1. Introduction

Postoperative nausea and vomiting (PONV) is defined as a postoperative gastrointestinal dysfunction, with mild PONV documented to have a negative impact on nutritional intake and comfort, and severe PONV leading to water-electrolyte disturbances, wound rupture, aspiration risk, and aspiration pneumonia [1]. It has a certain detrimental effect on postoperative recovery, and further takes a toll on patients' health and medical expenditure [2]. The incidence of PONVs induced by various surgeries is estimated to be 15%–46.1% [3, 4]. Postoperative nausea and vomiting is most commonly triggered by anesthesia, which has a depressing effect on nerve function, and in some cases may affect nerve function of the gastrointestinal tract, leading to nausea and vomiting [5]. Another predisposing factor is that if the patient is undergoing surgery on the gastrointestinal region, postoperative nausea and vomiting may also be triggered by damage to the gastric mucosa caused by surgical equipment during the procedure [6]. Postoperative nausea and vomiting are also likely to occur if postoperative care is inadequate and the diet is not observed [7].

The use of Western antiemetics is often associated with adverse reactions. Constipation is the most common adverse effect of 5-HT_3_ receptor antagonists, mainly due to reduced intestinal fluid secretion and slowed bowel movements caused by antiemetic drugs [8]. In addition, chemotherapeutic agents (e.g., vincristine) that interfere with gastrointestinal function and others such as impaired cortical function, impaired consciousness, and autonomic dysfunction can cause constipation [9]. Headache is also a common adverse effect of 5-HT_3_ receptor antagonists and NK-1 receptor antagonists, with the majority of patients experiencing mild dizziness and headache that resolves on its own [10].

Chinese medicine treatment for PONV has many advantages such as high safety, few adverse effects, and many targets, and therefore research on it has increased considerably. The PEG needle combines the advantages of traditional acupuncture and buried needles. The shallow stabbing and long retention of needles prolong the stimulation brought about by needling, increase the response to needling, promote the harmonious coexistence of breath power and blood in the meridians or internal organs, balance yin and yang, and work. It plays an important role in improving nausea and vomiting [11, 12]. Chinese medicine ironing therapy (Reyan bag) is an external treatment for patients under the guidance of the basic theories of TCM. By increasing the temperature of the covered area and acupuncture points, blood circulation is accelerated and drug absorption is increased, allowing for efficient local drug delivery [13].

This study was undertaken to assess and analyze the clinical efficacy of thumbtack needle therapy combined with Chinese medicine ironing therapy on PONV.

## 2. Materials and Methods

### 2.1. Baseline Data

One hundred and six patients who underwent surgery at our institution between January 2019 and December 2020 were selected for prospective analysis. The participants were randomly and equally divided into a control and an experimental group of 53 patients each. The study was approved by the Ethics Committee of the Zhuji Hospital of Traditional Chinese Medicine.

#### 2.1.1. Inclusion Criteria

1. Patients who received urological surgery
2. American Society of Anesthesiologists (ASA) grade I–III
3. Patients with no contraindications to general anesthesia

#### 2.1.2. Exclusion Criteria

1. Patients with nausea and vomiting caused by intracranial hypertension, gastrointestinal obstruction, and other reasons
2. Patients with mental disorders, mental retardation, consciousness disorders, and aphasia
3. Patients with a gastric tube after operation
4. Patients fainted on acupuncture or patients with skin injury, papules, skin swelling, and skin infection in the treatment location
5. Patients with allergy to treatment drugs

### 2.2. Intervention Methods

The control group was given normal modern medication to prevent and treat nausea and vomiting after general anesthesia. The experimental group was given thumbtack needle therapy combined with Chinese medicine ironing therapy to intervene nausea and vomiting after general anesthesia. The specific measures are as follows.

The Neiguan point (PC 6) and Zusanli point (ST 36) were selected. Disposable sterile needles were utilized and the locations where the needles were buried were disinfected with conventional iodophors. Then, forceps were used to clamp the handle and remove the medicinal adhesive cloth. Next, needles were pierced into the acupoints vertically. During needle retention, the needle-twirling therapy was discontinuously performed with moderate intensity, with about 4–5 min per time and an interval of 4 h. The herbal combination of the medicinal evodia fruit, Semen Raphani, Fructus Aurantii, Cortex Magnoliae Officinalis, and Fructus Foeniculi was used to make a hot herbal bag and placed in a microwave oven and heated to 40–45°C. During treatment, the patient was assisted to lie on his back, the abdomen was compressed with a Reyan bag, and the abdomen was push-pressed clockwise to the Tianshu points on both sides, 30 min per time, 3–4 times a day.

### 2.3. Observation Indicators

1. The score and incidence of PONV of patients at various time points after operation were recorded [14]. The score was rated according to the WHO criteria: 0 points: no nausea and vomiting; 1 point: no vomiting, but slight nausea and abdominal discomfort; 2 points: mild vomiting; 3 points: severe vomiting being difficult to control by medication; 4 points: intractable vomiting. Number of people with PONV/total number of people ×100% = PONV incidence.
2. The blood samples of patients were collected at 12 h and 48 h after operation for detection. Motilin, gastrin, and ghrelin were detected using enzyme-linked immunosorbent assay, which was in strict accordance with the kit instructions.
3. The FLIE was used to assess the patient's quality of life [15], with a total score ranging from 18 to 126 points. Higher scores indicate a better quality of life.
4. Kolcaba's GCQ scale was used to assess the patient's comfort [16], totaling 28 items in 4 dimensions of physiological, psychological, socio-cultural, and environmental. The full score is 112 points, and a higher score indicates greater comfort.

### 2.4. Statistical Analysis

Statistical analysis in the present study was done using SPSS20.0 software. The measurement data with normal distribution and homogeneity variance were expressed as *x* ± *s*. The *t*-test was carried out to examine the differences between the groups. Data that did not conform to normal distribution were presented as mean, and the differences were investigated using the Mann–Whitney *U* nonparametric test. The *X*^2^ test was employed for count data comparison. Significance was claimed at *P* value <0.05.

## 3. Results

### 3.1. Baseline Data

There were 33 males and 20 females in the control group, aged from 35 to 73 years (mean, 53.32 ± 4.37), and the average body mass index (BMI) was 22.37 ± 5.29 kg/m^2^. There were 29 males and 24 females in the experimental group, aged from 32 to 75 years (mean, 52.89 ± 5.19), and the average BMI was 22.69 ± 5.81 kg/m^2^. The baseline information of the two groups was homogenous.

### 3.2. Comparison of PONV Scores at Various Postoperative Time Points

The control group had a PONV score of 3.38 ± 0.82 at 0–6 h postoperative, 3.52 ± 0.77 at 6–12 h postoperative, 3.07 ± 0.81 at 12–24 h postoperative, and a mean score of 0.68 at 24–48 h postoperative; the experimental group had a PONV score of 2.52 ± 0.61 at 06 h postoperative, 6–12 h postoperative score was 2.59 ± 0.68, the score at 12–24 h after surgery was 2.23 ± 0.72, and the mean score at 24–48 h postoperative was 0. The score of PONV in the experimental group was found to be remarkably lower when compared against the control group at various time points (*P* < 0.05, Table 1).

### 3.3. Comparison of the Incidence of PONV at Various Postoperative Time Points

The incidence of PONV in the control group was 41.5% at 0–6 h postoperatively, 47.2% at 6–12 h postoperatively, 34.0% at 12–24 h postoperatively, and 9.4% at 24–48 h postoperatively; the incidence of PONV in the experimental group was 17.0% at 0–6 h postoperatively, 20.8% at 6–12 h postoperatively, 12–24 h postoperatively incidence of 11.3%, and 0% for 24–48 h postoperatively.  Table 2 shows that the incidence of PONV in the experimental group was lower than that of control group at various postoperative time points (*P* < 0.05).

### 3.4. Changes in Gastrointestinal Hormone Levels before Operation and 12 h and 48 h after Operation

The *t*-test showed that gastrointestinal hormone levels of the experimental group were higher than those of the control group at 12 h and 48 h after operation, and the differences were completely significant (*P* < 0.05, Table 3).

### 3.5. Comparison of Comfort between the Two Groups before Operation, 24 h and 48 h after Operation

In the control group, the postoperative comfort level was 65.72 ± 12.65 points at 24 h and 78.23 ± 15.29 points at 48 h; in the experimental group, the postoperative comfort level was 81.63 ± 15.87 points at 24 h and 95.21 ± 18.96 points at 48 h. A statistically significant difference in the comparison in GCQ between the experimental group and the control group was noticed, as shown in Table 4.

### 3.6. Comparison of the Quality of Life between the Two Groups

In the control group, the quality of life score was 75.31 ± 15.62 at 24 h and 87.96 ± 17.62 at 48 h after surgery; in the experimental group, the quality of life score was 93.27 ± 18.85 at 24 h and 107.68 ± 20.28 at 48 h after surgery. On overall assessment, a significant increase was seen in the scores of the FLIE of the experimental group (*P* < 0.05, Table 5).

## 4. Discussion

The mechanism of PONV is currently unclear and is presumed to be related to a combination of the patient's own factors, anesthesia, and surgery-related risk factors [17]. Although common antiemetics are often used after surgery to reduce the incidence of PONV, they still face the challenges of grim outcomes, high economic costs, and side effects in many ways. To date, there is no specific treatment for PONV, which is usually prevented and treated through medical care interventions.

TCM categorizes nausea and vomiting to the “vomiting” field, and believes that the PONV is caused by the invasion of pathogenic factors and deficiency of the healthy breath power, further leading to the disorders of breath power in Zhang-fu organs and the stasis of breath power and blood as well as stagnation in meridians. Subsequently, the disturbance in ascending and descending in San jiao (triple energizer) gasification and adverse rising of stomach breath power arises. The disease is mainly located in the spleen and the stomach. The mechanism is considered to be derived from the disorder of the spleen and the stomach, and adverse rising of stomach breath power. The treatment principle thus should be based on regulating the flow of breath power, harmonizing the stomach, and descending adversely risen stomach breath power to stop vomiting [18]. A growing body of evidence confirms the great potential of acupuncture for digestive motility, secretion, and absorption to improve the quality of postoperative analgesia, promote recovery of postoperative gastrointestinal function, and reduce the incidence of PONV [19, 20]. Thumbtack needling therapy is a type of floating or shallow stabbing in traditional acupuncture to promote the circulation of breath power and blood in the meridian defence. Additionally, it can also nourish the defensive yang by needle retention. Thus, the thumbtack needling therapy might treat the symptoms and the root cause simultaneously, to invigorate breath power, promote blood circulation, activate collaterals, and relieve pain. From the perspective of modern medicine, it is contributed to mild and persistent stimulation on nerve terminal receptors and central nerves to inhibit pathological excitement, and improve body reaction [21].

The Neiguan point (PC 6) is the main point to stop vomiting. It has an excellent regulating effect on the blood circulation, digestive system, and endocrine system. More importantly, it also activates the body's immune surveillance and improves the body's immune function. Significantly, it acts on the vomiting centre in the medulla oblongata to suppress the onset of nausea and vomiting [22]. The Zusanli point (ST 36) has the function of regulating the spleen and the stomach, regulating breath power and blood, governing digestion, and tonifying weakness. The combination of the Neiguan point (PC 6) and the Zusanli point (ST 36) could regulate the flow of breath power and restore breath power, harmonize the stomach and reduce adverse reactions, and improve PONV. This therapy fully embodies TCM ideas [23]. The studies of Sun yun have demonstrated that the treatment of thumbtack needles at the Neiguan point and the Zusanli point can effectively improve nausea and vomiting symptoms of patients after chemotherapy with colorectal cancer. The medicinal evodia fruit has the effects of warming meridians to dissipate cold, descending adversely risen stomach breath power to stop vomiting, reinforcing yang and alleviating diarrhea, and is mainly used for stomach pain, nausea, and vomiting. Fructus aurantii and Cortex Magnoliae Offcinalis are the main herbs to regulate the flow of breath power and relieve distension, promote the vomit efficacy of dampness retained in middle energizer, and retention of food in the stomach. Foeniculi has the functions of dissipating cold to kill pain and regulating the flow of breath power and harmonizing the breath power of the stomach, and is mainly used for the abdominal cold pain. The Chinese medicine ironing (Reyan bag) is used after being heated to make the striated layer loose, promote the penetration and absorption of drugs, balance breath power and blood, yin and yang, adjust the function of zang-fu organs, and improve the physiological process of the patient in general [24, 25]. This study showed that the score and incidence of PONV in the experimental group were lower than those in the control group, indicating that the intervention of thumbtack needles and embedding needles therapy combined with Chinese medicine ironing therapy plays a positive role in PONV, which can significantly improve the symptoms of nausea and vomiting and reduce the incidence of PONV. It can be served as an alternative clinically.

Prior thumbtack needling therapies have shown that gastrointestinal system regulation and body fluids play a key role in gastrointestinal recovery [26]. Gastrointestinal hormones regulate gastrointestinal movement through the endocrine system, cavity secretion, and the excitation or/and inhibition of neurotransmitters. Gastrointestinal functional activities are inhibited after operation, resulting in the decrease of motilin, gastrin, and ghrelin levels [27]. The findings of this study revealed that the level of the gastrointestinal hormone in the experimental group was observed to be comparatively higher after treatment compared to that in the control group. The possible explanation is that this technique increases angiotensin, promotes gastrointestinal peristalsis, and accelerates the recovery of the gastrointestinal hormone, thus reducing PONV. Huang et al. (2015) suggested that acupuncture can regulate gastrointestinal hormone secretion, reduce the inhibition of gastrointestinal digestion function, and promote the recovery of gastrointestinal movements [28].

The present study showed that a significantly better quality of life and comfort of patients in the experimental group were noticed. It is presumably because the technique is characterized by easy operation, quick effectiveness and less pain, and movement-friendly. The collaboration of the two together is conducive to improve the symptoms of PONV, the comfort, and quality of life of patients.

There are certain flaws in our experiment. First of all, because the sample size is too small, there will inevitably be a chance for errors. Second, we need to conduct more detailed research on postoperative antiemetics of different disease types in subsequent experiments to establish a more detailed classification.

## 5. Conclusion

To conclude, 0–12 h after operation may be the peak stage of PONV under general anesthesia. Thus, we recommend thumbtack needling combined with Chinese herbs ironing as a preferred option due to its benefits in relieving discomfort, reducing the incidence of PONV, and improving the level of gastrointestinal hormones and enhancing the quality of patients.

## Figures and Tables

**Table 1:** Comparison of PONV scores between the two groups of patients at various postoperative time periods ($\bar{X}$ ± *s*, score, *n* = 53).

Group	0–6 h	6–12 h	12–24 h	24–48 h (mean)
Control group	3.38 ± 0.82	3.52 ± 0.77	3.07 ± 0.81	0.86
Experimental group	2.52 ± 0.61	2.59 ± 0.68	2.23 ± 0.72	0
*t*	6.126	6.591	5.643	9.632
*P*	≤0.001	≤0.001	≤0.001	≤0.001

**Table 2:** Comparison of the incidence of PONV between the two groups of patients at various time periods after operation (*n*, %, *n* = 53).

Group	0–6 h	6–12 h	12–24 h	24–48 h
Control group	22 (41.5)	25 (47.2)	18 (34.0)	5 (9.4)
Experimental group	9 (17.0)	11 (20.8)	6 (11.3)	0 (0)
*χ* ^2^	7.705	8.244	7.756	5.248
*P*	0.006	0.004	0.005	0.022

**Table 3:** Changes of gastrointestinal hormone levels before operation and 12 h and 48 h after operation.

Group		24 h after operation	48 h after operation
Control group	Gastrin	47.26 ± 9.73	54.59 ± 11.67
	Motilin	76.29 ± 11.62	87.93 ± 10.85
	Ghrelin	83.78 ± 13.62	97.65 ± 15.97

Experimental group	Gastrin	76.55 ± 12.66^*∗*^	83.22 ± 15.62^*∗*^
	Motilin	119.82 ± 18.76^*∗*^	131.28 ± 20.52^*∗*^
	Ghrelin	125.62 ± 19.36^*∗*^	153.26 ± 23.75^*∗*^

**Table 4:** Comparison of comfort between the two groups before operation, 24 h and 48 h after operation ($\bar{X}$ ± *s*, score, *n* = 53).

Group	24 h after operation	48 h after operation
Control group	65.72 ± 12.65	78.23 ± 15.29
Experimental group	81.63 ± 15.87	95.21 ± 18.96
*t*	5.141	9.528
*P*	≤0.001	≤0.001

**Table 5:** Comparison of the quality of life between the two groups ($\bar{X}$ ± *s*, score, *n* = 53).

Group	24 h after operation	48 h after operation
Control group	75.31 ± 15.62	87.96 ± 17.62
Experimental group	93.27 ± 18.85	107.68 ± 20.28
*t*	5.341	5.344
*P*	≤0.001	≤0.001

## Data Availability

All data generated or analysed during this study are included in this published article.

## References

[1] Islam S., Jain P. N. (2004). Post-operative nausea and vomiting (PONV): a review article. *Indian Journal of Anaesthesia*.

[2] Talebpour M., GhiasnejadOmrani N., Imani F., Shariat Moharari R., Pourfakhr P., Khajavi M. R. (2017). Comparison effect of promethazine/dexamethasone and metoclopramide /dexamethasone on postoperative nausea and vomiting after laparascopic gastric placation: a randomized clinical trial. *Anesthesiology and Pain Medicine*.

[3] Dobbeleir M., De Coster J., Coucke W., Politis C. (2018). Postoperative nausea and vomiting after oral and maxillofacial surgery: a prospective study. *International Journal of Oral and Maxillofacial Surgery*.

[4] Gouveia de Araujo Ferreira N., Cavalcanti I. L., Assad A. R., Barrucand L., Braga E. L. C., Verçosa N. (2020). A prospective, randomized, double-blind trial to compare body weight-adjusted and fixed doses of palonosetron for preventing postoperative nausea and vomiting in obese female patients. *PLoS One*.

[5] Shaikh S. I., Nagarekha D., Hegade G., Marutheesh M. (2016). Postoperative nausea and vomiting: a simple yet complex problem. *Anesthesia: Essays and Researches*.

[6] Kehlet H. (1997). Multimodal approach to control postoperative pathophysiology and rehabilitation. *British Journal of Anaesthesia*.

[7] Kenny G. N. C. (1994). Risk factors for postoperative nausea and vomiting. *Anaesthesia*.

[8] Wolf H. (2000). Preclinical and clinical pharmacology of the 5-HT3 receptor antagonists. *Scandinavian Journal of Rheumatology*.

[9] Morgillo A., Marovino E. (2021). Chemotherapy neurotoxicity: pharmacological and toxicological aspects. *International Journal of Current Research*.

[10] Navari R. M. (2015). 5-HT3 receptors as important mediators of nausea and vomiting due to chemotherapy. *Biochimica et Biophysica Acta (BBA)-Biomembranes*.

[11] Hu C., Gong L., Zhang B. (2019). Clinical observation of acupoint pressing needle combined with western medicine in the prevention and treatment of chemotherapy-related nausea and vomiting of small cell lung cancer. *Shanghai Journal of Acupuncture*.

[12] Liang F., Ma Y., Liu H. (2019). Research progress on the main clinical application of press needle. *Journal of Traditional Chinese Medicine*.

[13] Ming D. M., Li C. W., Hui D. Y. (2019). A brief introduction to the recent clinical application of traditional Chinese medicine reyanbao. *Jiangxi Traditional Chinese Medicine*.

[14] Weilbach C., Rahe-Meyer N., Raymondos K., Weissig A., Scheinichen D., Piepenbrock S. (2006). Postoperative nausea and vomiting (PONV): usefulness of the apfel-score for identification of high risk patients for PONV. *Acta Anaesthesiologica Belgica*.

[15] Martin A. R., Pearson J. D., Cai B. (2003). Assessing the impact of chemotherapy-induced nausea and vomiting on patients’ daily lives: a modified version of the functional living index-emesis (FLIE) with 5-day recall. *Supportive Care in Cancer*.

[16] Zhang Y., Hou R., Li Y. (2017). Research progress of comfort measurement tools. *Journal of Nursing*.

[17] Yang S., Yang L., Zheng W. (2017). Research progress on prevention and treatment of postoperative nausea and vomiting. *Practical Medicine and Clinical*.

[18] Li C., Li H., Chen T. (2017). Study on the preventive and therapeutic effect of transcutaneous acupoint electrical stimulation on nausea and vomiting after craniotomy tumor resection. *China Emergency of Traditional Chinese Medicine*.

[19] Yin Z., Xiao Q., Xu G. (2020). Acupuncture for the postcholecystectomy syndrome: a systematic review and meta-analysis. *Evidence-Based Complementary and Alternative Medicine*.

[20] An L.-X., Chen X., Ren X.-J., Wu H.-F. (2014). Electro-acupuncture decreases postoperative pain and improves recovery in patients undergoing a supratentorial craniotomy. *The American Journal of Chinese Medicine*.

[21] Qi S., Ning L. (2019). History and mechanism of press needle. *Clinical Research of Traditional Chinese Medicine*.

[22] Zhu Y. (2019). Clinical application of neiguan point in prevention and treatment of postoperative nausea and vomiting. *Clinical Research of Traditional Chinese Medicine*.

[23] Wu F. Z., pan H. Y., Wang Z. (2020). Analysis of acupoint selection of postoperative nausea and vomiting patients based on data mining. *Nursing Research*.

[24] Sun Y., Duan Y., Bai X. (2019). Effect of pressing needle and embedding needle on alleviating nausea and vomiting in patients with colorectal cancer after chemotherapy. *Nursing of Integrated Traditional Chinese and Western Medicine (Chinese and English)*.

[25] Zhang J. (2016). Application of traditional Chinese medicine reyanbao combined with ironing therapy in patients with cold and qi stagnation stomachache. *Nursing Research*.

[26] Liu C., Fang X., Wang T. (2019). Effect of midnight noon ebb flow on gastrointestinal function recovery after gynecological laparoscopic surgery. *Journal of Modern Integrated Traditional Chinese and Western Medicine*.

[27] Hou L., Xu L., Shi Y. (2016). Effect of electric acupoint stimulation on gastrointestinal hormones and motility among geriatric postoperative patients with gastrointestinal tumors. *Journal of Traditional Chinese Medicine*.

[28] Huang L., Yu Q., pan J. F. (2015). Effect of acupuncture on gastrointestinal function recovery and gastrointestinal hormone secretion after abdominal surgery. *Journal of Anhui University of Traditional Chinese Medicine*.

